RETRACTED

# Research on Keyword Extraction Algorithm in English Text Based on Cluster Analysis

**DOI:** 10.1155/2022/4293102

**Published:** 2022-03-28

**Authors:** Jingxia Ma

**Affiliations:** School of Western Languages and Cultures, Harbin Normal University, Harbin 150025, China

## Abstract

How to facilitate users to quickly and accurately search for the text information they need is a current research hotspot. Text clustering can improve the efficiency of information search and is an effective text retrieval method. Keyword extraction and cluster center point selection are key issues in text clustering research. Common keyword extraction algorithms can be divided into three categories: semantic-based algorithms, machine learning-based algorithms, and statistical model-based algorithms. There are three common methods for selecting cluster centers: randomly selecting the initial cluster center point, manually specifying the cluster center point, and selecting the cluster center point according to the similarity between the points to be clustered. The randomly selected initial cluster center points may contain “outliers,” and the clustering results are locally optimal. Manually specifying the cluster center points will be very subjective because each person's understanding of the text set is different, and it is not suitable for the case of a large number of text sets. Selecting the cluster center points according to the similarity between the points to be clustered can make the selected cluster center points distributed in each class and be as close as possible to the class center points, but it takes a long time to calculate the cluster centers. Aiming at this problem, this paper proposes a keyword extraction algorithm based on cluster analysis. The results show that the algorithm does not rely on background knowledge bases, dictionaries, etc., and obtains statistical parameters and builds models through training. Experiments show that the keyword extraction algorithm has high accuracy and can quickly extract the subject content of an English translation.

## 1. Introduction

With the advancement of information technology, mankind is carrying out the biggest project in the history of information on the Internet, and at the same time, there is also a constant stream of new information being produced on the Internet. Anyone can publish any information through the network at any time and any place [1, 2]. The entire web is piling up into an unprecedented super-large database, which means that the web has become a huge and disorganized desktop library. Facing the flood of electronic documents, people urgently need various online intelligent services that can automatically collect, filter, organize, and utilize information. Information retrieval, automatic summarization, text clustering/classification, and topic search are all very powerful intelligent tools [3–5].

RETRACTED

When people are browsing through English texts, news with valuable content but not enough headlines is easy to ignore. Furthermore, it is difficult to determine the desired target information only from the vague generalizations retrieved. An effective way to solve these problems is to give the keywords of the text. As a brief summary of the content of the article, keywords can help people quickly understand the main content of the article and save browsing time. In addition, keywords also play a large role in the fields of information retrieval, automatic summarization, text clustering/classification, and topic search [6–9]. However, many news web pages on the Internet currently do not have keywords, and selecting keywords manually is time-consuming and highly subjective. Therefore, automatic keyword extraction from content has become an important topic.

Many researchers have conducted in-depth research on the keyword extraction algorithm and cluster center point selection algorithm in the process of text clustering so as to optimize the clustering results. There are many existing keyword extraction algorithms, which can be divided into three categories: algorithms based on statistical models, algorithms based on semantics, and algorithms based on machine learning [10–12]. The traditional clustering algorithm in Euclidean space selects the initial cluster center point in a random way and iteratively updates the cluster and the cluster center point so that the cluster center point is getting closer and closer to the class center point, but due to the initial cluster center point. The number and location of the clustering center points are random, and the clustering results may appear to be locally optimal. Therefore, many scholars have devoted themselves to the research of the clustering center point selection algorithm, and a variety of clustering center point selection algorithms have appeared. This method is suitable for text clustering algorithms, optimizing clustering results and extracting keywords [13–16].

There are two common ways to select cluster center points: one is to randomly select *k* initial cluster center points, and the other is to select cluster center points according to a certain measurement method. The method of randomly selecting initial cluster center points is suitable for clustering in traditional Euclidean space [17–20]. For the same test data set, the initial cluster center points randomly selected each time are different, the results of assigning the to-be-clustered points to the clusters and iteratively updating the cluster and cluster center points are different, and the final clustering results are also different. A local optimum occurs. In this method, although the initial center points are randomly selected, after repeated updates, the obtained cluster center points have a high density, although the number of initial cluster center points is randomly selected. The number of obtained cluster center points is consistent with the number of initial cluster center points, so objects belonging to the same class will be divided into multiple classes, or objects belonging to multiple classes will be assigned to one class, and finally, this leads to the local optimum of the clustering results [21–23]. The method of selecting the cluster center point according to a certain measurement method is suitable for text clustering. After this method selects the cluster center point, the text is assigned to the cluster where the center point with the greatest similarity is located; that is, the text clustering is completed [24, 25]. There is no iterative update process for the selected center points, so the selection of cluster center points is very important. The ideal cluster center point should be scattered in each class, close to the class center point, with high density, and there should be no “isolated point” in it, the cluster obtained after text clustering according to the selected cluster center point, the texts within the clusters have the largest similarity, and the clusters have the smallest similarity. The common method for selecting the cluster center point for text clustering is to select the cluster center point by calculating the similarity between the texts. Points that are correlated with more texts are used as cluster center points, and so on [26–29].

RETRACTED

The existing keyword extraction algorithms under text include semantic-based keyword extraction algorithms, which rely on background knowledge bases, dictionaries, vocabulary lists, etc., and cannot extract words or phrases that are not included in the knowledge base; machine learning-based keywords and phrases cannot be extracted [30–32]. The word extraction algorithm depends on the selected algorithm model, and the training takes a long time; the keyword extraction algorithm based on the statistical model has a simple principle, does not require training samples, and does not depend on the knowledge base. Many scholars have devoted themselves to the research of cluster center point selection algorithms in text clustering. Common cluster center point selection is based on the similarity between texts. For example, points that are far away from each other are used as clusters. The method of the center point, the method of selecting the point that has correlation with more points to be clustered as the center point of the cluster, and the method of selecting the point with greater similarity with the points to be clustered as the center point of the cluster, all wait. The purpose of using these methods is to hope that the selected cluster center points are distributed in each class and are close to the class center points [4, 33–35].

In this work, we mainly explore keyword extraction based on cluster analysis. By analyzing and comparing four kinds of commonly used keyword extraction algorithms: statistical information method, structure-based method, natural language understanding-based, and machine learning-based method, and comprehensively utilizing the advantages of cluster analysis, a training-independent method is proposed. It is not only effective and feasible, but also makes up for the lack of mechanical statistical methods by analyzing the important words in the text from the perspective of semantics. At the same time, the limitations faced by machine learning methods and the lack of annotated corpora are eliminated [9–11, 36].

The structure of this paper is arranged as follows: the first chapter mainly introduces the research significance and the theoretical basis of the technology; the second chapter introduces the linguistic background of keyword extraction technology and its application in keyword extraction and introduces the main clustering analysis methods and its advantages and disadvantages. The third chapter combines the shortcomings of existing keyword extraction algorithms and the advantages of hierarchical clustering algorithms to build hierarchical clustering, describes its implementation process in detail and compares the experimental results with traditional mechanical statistical methods. The fourth chapter presents the experimental data of an example and the test results of a large-scale corpus. The fifth chapter mainly summarizes the paper and proposes the next task [11, 13].

The research contributions of the paper include the following:

1. This paper introduces three clustering processing methods, such as randomly selecting the initial cluster center point, manually specifying the cluster center point, and according to the points to be clustered.
2. This paper proposes a keyword extraction algorithm based on cluster analysis.
3. The algorithm proposed in the paper shows that the algorithm does not rely on background knowledge bases, dictionaries, etc., and obtains statistical parameters and builds models through training.

## 2. Keyword Extraction Background and Related Work

### 2.1. Keyword Concept

Keywords are considered to be a collection of the most important and semantically similar words in an article. Clustering is the dividing of a set of data units into several subsets called “clusters” or “categories.” The data in each category has similarities, and its division is based on “clustering of objects.” The basis of clustering according to the distance between points is that distance is a logical concept, indicating the similarity between points. Therefore, this paper uses the relationship between words and adopts the clustering method to extract the most important keywords that have a great relationship with the theme according to the principle of the similarity of the theme [14, 16, 17, 37]. Keywords are words or terms used to express the subject content, information, and entries of the article: it is a noun term reflecting the content of the article; it is extracted from the title, abstract, hierarchical title, and solicitation of the article, and has substantial meaning to the content of the article. A word or phrase is a natural language vocabulary that expresses the subject concept of a document. In terms of form, keywords or concepts are words that appear in the title, abstract, and text of the article and are the words or proper nouns of the author; in terms of content, keywords or concepts should have specific meanings and reflect specific concepts. The real words or phrases of the text can be terms of various professions, such as computer, network, automobile, natural language understanding, information system, etc., or can be proper nouns, such as Beijing, Shanghai, Iraq, Bush, People's Daily, etc.; in terms of function, it can express the subject content of the article. The quality of keywords is closely related to the content of each point of the article. Therefore, to effectively extract keywords, it is necessary to fully understand the content of the article and the exact meaning of each word in the article. An article is not just a collection of words, but there is a theme of the article expressed by many words hidden beneath the surface. The understanding of the words in the text cannot be isolated, and the words that are semantically similar or closely related in the text should be linked together.

RETRACTED

### 2.2. Cluster Analysis

The basic feature of the cluster analysis problem is to classify some objects with similar attributes into the same set; that is, when the dataset is analyzed, the class labels of the objects in the training data are unknown, and we can generate them by clustering. The generation of class labels relies on the law of “maximizing the similarity of objects within a class and minimizing the similarity of objects between classes” to form clusters of objects. The dissimilarity is an important measure to distinguish the similarity between data and between classes, and its calculation is based on the attribute value of the described object. Distance is a measure that is often used. Based on the introduction of the concept and application of clustering and its typical requirements for clustering algorithms, this chapter introduces the data structure required for dissimilarity calculation and details how to calculate the distance between objects represented by various attributes and types. Finally, the cluster analysis method is briefly analyzed and discussed.

**Basic data structure:** it describes *n* objects with *p* variables, such as age, height, gender, race, etc. to describe the object “person”. It can be defined as an *n*∗*p*-dimensional matrix.

(1) $$\begin{array}{c} \left[\begin{array}{ccccc} x11 & \cdots & x1f & \cdots & x1p\\ \vdots & \vdots & \vdots & \vdots & \vdots \\ xi1 & \cdots & \text{xif} & \cdots & \text{xip}\\ \vdots & \vdots & \vdots & \vdots & \vdots \\ xn1 & \cdots & \text{xnf} & \cdots & \text{xnp} \end{array}\right]. \end{array}$$

Dissimilarity matrix stores the approximation between *n* objects, expressed as an *n*∗*n*-dimensional matrix.

(2) $$\begin{array}{c} \left[\begin{array}{ccccc} 0 & \; & \; & \; & \;\\ d\left(2,1\right) & 0 & \; & \; & \;\\ d\left(3,1\right) & d\left(3,2\right) & 0 & \; & \;\\ \vdots & \vdots & \vdots & 0 & \;\\ d\left(n,1\right) & d\left(n,2\right) & \cdots & \cdots & 0 \end{array}\right]. \end{array}$$

Conversely, the more dissimilar the two objects are, the larger their value will be. It is converted to a dissimilarity matrix before using this type of algorithm.

The selected unit of measure will directly affect the results of the cluster analysis. For example, changing the unit of measure for height from “meters” to “feet” or for the weight from “kilograms” to “pounds” may result in very different clustering structures. How to normalize the data of a variable? In order to achieve standardization of measures, one method is to shift the original measure to a value. Given a measure *f*, the transformation can be shown as follows:

(3) $$\begin{array}{c} Sf=\frac{\left(\left|X_{1f}-m_{f}\right|+\left|X_{2f}-m_{f}\right|+\cdots +\left|X_{nf}-m_{f}\right|\right)}{n}. \end{array}$$

In which, Xif is the different measurement values of *f*, and mf represents the average of *f*, which is specifically expressed as follows:

(4) $$\begin{array}{c} m_{f}=\frac{\left(X_{1f}+X_{2f}+\cdots +X_{nf}\right)}{n}. \end{array}$$

We calculate the normalized measure, or z-score as the following formula:

(5) $$\begin{array}{c} Zi_{f}=\frac{\left(X_{\text{if}}-m_{f}\right)}{S_{f}}. \end{array}$$

“The data has been normalized, how to calculate the dissimilarity between objects?” After normalization, or in some applications without normalization, it will be calculated as follows:

(6) $$\begin{array}{c} d\left(i,j\right)=\sqrt{{\left|x_{i1}-x_{j1}\right|}^{2}+{\left|x_{i2}-x_{j2}\right|}^{2}+\cdots +{\left|x_{ip}-x_{jp}\right|}^{2}}. \end{array}$$

Here the Manhattan distance between *x*_i_ and *x*_j_ will be defined as follows:

(7) $$\begin{array}{c} d\left(i,j\right)=\left|x_{i1}-x_{j1}\right|+\left|x_{i2}-x_{j2}\right|+\cdots +\left|x_{\text{ip}}-x_{\text{jp}}\right|. \end{array}$$

Minkowski Distance is defined as follows:

(8) $$\begin{array}{c} d\left(i,j\right)=\sqrt[{q}]{{\left|x_{i1}-x_{j1}\right|}^{q}+{\left|x_{i2}-x_{j2}\right|}^{q}+\cdots +{\left|x_{\text{ip}}-x_{\text{jp}}\right|}^{q}}. \end{array}$$

If each variable is given a weight according to its importance, the weighted Euclidean distance can be calculated as follows:

(9) $$\begin{array}{c} d\left(i,j\right)=\sqrt{w_{1}{\left|x_{i1}-x_{j1}\right|}^{2}+w_{2}{\left|x_{i2}-x_{j2}\right|}^{2}+\cdots +w_{p}{\left|x_{\text{ip}}-x_{\text{jp}}\right|}^{2}}. \end{array}$$

For example, given a variable describing a patient as a smoker, 1 means the patient smokes, and 0 means the patient does not. Treating binary variables like interval-scaled variables can mislead clustering results, so specific methods are used to calculate their dissimilarity. When some or all binary variables are encoded, the calculation result will not change. For constant similarity, the most well-known simple matching coefficient between two objects *i* and *j* is defined as follows:

(10) $$\begin{array}{c} d\left(i,j\right)=\frac{r+s}{q+r+s+t}. \end{array}$$

Therefore, such binary variables are often thought of as having only one state. Similarities based on such variables are called non-constant similarities. For nonconstant similarity, the most well-known evaluation coefficient is the Jaccard coefficient, in which the number of negative matches is considered unimportant and therefore ignored.

(11) $$\begin{array}{c} d\left(i,j\right)=\frac{r+s}{q+r+s}. \end{array}$$

When both symmetric and asymmetric binary variables are present in the same dataset, the mixed-variables approach can be applied.

RETRACTED

## 3. Research Status of Keyword Extraction Technology

There are three main evaluation conferences for information extraction: MUC (message understanding conference), MET (multilingual entity task conference), and TREC (text retrieval conference). Among them, MUC is a regular conference supported by the US government dedicated to the understanding of real news texts. In addition to exchanging papers like a general academic conference, it is also responsible for organizing a series of evaluation activities for message understanding systems from different units around the world. Its main evaluation project is to extract specific information from news reports and fill it into some kind of database. Most of the evaluation corpus comes from news released by major news agencies. For each message, a standard answer is given manually by professionals, and then the output results of the participating systems are compared with the standard answers, and the evaluation results of all systems are given according to certain evaluation indicators. The most important indicators are the accuracy rate, recall rate, etc. Currently, the concepts, models, and technical specifications defined by MUC play a leading role in the entire field of information extraction internationally.

In information extraction, the recall rate can be described as the ratio of correctly extracted information; that is, how much information is extracted correctly, while the accuracy rate can be described as the correct ratio of the extracted information, that is, the credibility of the extracted information. The specific definitions are as follows:

(12) $$\begin{array}{c} \text{precision}=\frac{\text{extraction\_correct\_keywords}}{\text{extraction\_keywords}}\text{,}\\ \text{recall}=\frac{\text{extraction\_correct\_keywords}}{\text{overall\_correct\_keywords}}\text{.} \end{array}$$

The values of precision and recall are between 0 and 1 (the maximum is 1), and there is a balanced relationship; that is, when the recall rate is low, a higher accuracy rate can often be achieved; on the contrary, when the recall rate is high, the reverse is true. The accuracy is often lower. When comparing the performance of different information extraction systems, both recall and precision need to be considered. However, comparing the parameters of two indicators at the same time is not intuitive, so the method of combining the two indicators into one indicator is proposed, such as F1 is defined as follows:

(13) $$\begin{array}{c} Ft=\frac{2*R*P}{R+P}. \end{array}$$

Linguistic experts can manually extract satisfactory subject words from documents, but for massive document information, it is not advisable to rely on human experts to manually extract subject words, and this method cannot extract keywords from a large number of words. Statistical method count the frequency of each word in the document and use the word whose frequency is higher than a certain threshold as a keyword. Although this method is simple and fast, it ignores the importance of some high-frequency words and some relatively low-frequency words. Important but very high-level issues such as word frequency, word co-occurrence, complex network features, and other methods.

RETRACTED

## 4. English Keyword Extraction Algorithm Based on Hierarchical Clustering

Generally, the content is to describe an event that occurs at the moment, so these keywords are important. On the other hand, it pays too much attention to the frequency of occurrence of words, and in the iterative calculation process, it tends to assign higher frequency to words with higher frequency. The weight of the keywords that appear infrequently is easily missed. Therefore, this algorithm takes the semantic difference between words as the innovative breakthrough point. The ending weights of words are obtained by iterative calculation, and the keywords are obtained by sorting. The general process is shown in Figure 1.

As shown in the figure, the general steps are as follows:

(1) Text preprocessing such as word segmentation, sentence segmentation, and filtering stop words.
(2) Calculate the clustering importance of words. The specific method is to use the BERT model to generate a corresponding word vector for each word so that these word vectors can be used to replace the corresponding words for k-means clustering, and the clustering importance is assigned to the words according to the clustering results.
(3) Calculate the positional importance of the word according to the different positions of the word in the title and text.
(4) Compute the importance degree of edges according to the word importance obtained in the above steps, thereby constructing a new state transition matrix.
(5) According to this state transition matrix, the weight of the word is calculated by continuous iteration until it converges, and finally, the weight of the word is sorted to obtain the final keyword.
  (14) $$\begin{array}{c} WS\left(Vi\right)=\left(1-d\right)+d*\sum_{Vj\in In\left(Vi\right)}\frac{\text{wji}}{\sum_{vk\in \text{Out}\left(Vj\right)}\text{wjk}}WS\left(Vj\right). \end{array}$$

The iterative calculation needs to be conducted according to the following formula:

(15) $$\begin{array}{c} WS\left(Vi\right)=\left(1-d\right)+d*\sum_{Vj\in In\left(Vi\right)}p_{ji}*WS\left(Vj\right). \end{array}$$

Let *wij*/∑_*vk*∈*out*(*vj*)_*wjk* denote the transport probability of *j* to *i*, then formula (15) can be defined as follows:

For any word a in the Ci set, the clustering importance of word a can be defined by the following formula:

(16) $$\begin{array}{c} \text{wvec}\left(a\right)=\left\{\begin{array}{c} t,\overset{⟶}{a}\_\text{is}\_\text{centroid}\\ 1,\overset{⟶}{a}\_\text{is}\_\text{not}\_\text{centroid} \end{array}.\right. \end{array}$$

Where a represents the word vector corresponding to word a, and *t* is the preset weight and in our work is 6.

RETRACTED

Because the similarity threshold *T* is different, the corresponding complex network community division accuracy is different, and its F-Measure varies with the text-similarity threshold *T* as shown in Figure 2. By analyzing the experimental results of each data set in Figure 2, it can be seen that the clustering effect is best when the text-similarity threshold *T* is between 0.1 and 0.2. Similarly, we can randomly sample other datasets for experiments with roughly the same results. Therefore, we consider texts with a similarity threshold greater than 0.15 to be neighbor texts. For other datasets, we use the similarity threshold *T* of 0.15 to establish a network and divide them into communities. The result of text clustering is shown in Table 1.

The analysis of the test results shows that the clustering quality of this algorithm is improved compared with the traditional K-means clustering algorithm, and the algorithm based on complex network community division is also used to achieve text clustering. The extracted algorithm also improved the clustering quality. Extracting feature text to reduce the number of texts does not reduce the F-measure of clustering. On the contrary, there is a certain improvement. The clustering result can be used as a training sample for future text classification. 80% of the feature texts are extracted from the original text set, which means that the training text is reduced by 25%, which means that the calculation amount can be reduced by 30% in the future text classification. While improving the quality of text clustering, the algorithm is also very effective for keyword extraction.

The results in Figure 3 are analyzed by different models. By comparing the accuracy, recall, and Ft of different keyword extraction algorithms in Figure 3, it can be seen that compared with the other three keyword extraction algorithms, our method has a certain extraction accuracy. Compared with the text2 algorithm, the accuracy is increased by 10%, the text3 algorithm is increased by 1%, and the accuracy is increased by 20% compared with the text4 algorithm.

Figure 4 shows the extraction results of the top 15 keywords under the same text by random, AlchemyAPI, and our method. It can be seen from the figure that the comparison results of the three methods are different. From the experimental results, it can be found that the performance of our method is 30% higher than random and 5% higher than AlchemyAPI in terms of precision (1% and 0.5%). Our method also significantly outperforms other methods in terms of overall recall and precision. To sum up, the keyword extraction algorithm based on cluster analysis proposed in this paper can well solve the problem of keyword extraction in English text.

RETRACTED

## 5. Conclusion

Using the complex network theory, we propose a new method of weighted complex network community division to find the dense density in the complex network and operate it to achieve the purpose of the complex network community division. According to the relationship between texts, a weighted complex network can be formed, and the complex network is divided into communities by the method, which realizes the clustering of texts. According to the existing method of using a complex network to extract text keywords, we propose a new method for keyword extraction. The comprehensive eigenvalue calculation method shows a high degree of connectivity in the entire network and, at the same time, shows a high degree of aggregation in the local network, which can better reflect the text topic. The operation of text clustering and keyword extraction through the method of complex networks requires that the network composed of text should be a sparse network. The question of how to accurately set the threshold value so that the network formed is a sparse network is the focus of future research.

This paper mainly conducts in-depth research on the keyword extraction algorithm for a given text. The purpose of keyword extraction is to extract words or phrases from the text that can refer to the subject of the text; the purpose of clustering center point selection is to select the cluster center points that are distributed in each class and are close to the class center point and optimize the clustering result. In the following research work, we can pay attention to the following aspects: when extracting words or phrases, the keyword extraction algorithm in this paper simultaneously extracts the starting and ending position information of words or phrases in the text. Based on this, we can discuss this in-depth problems with word co-occurrence. Existing keyword extraction algorithms are generally applicable to one language, and it is possible to deeply study how to improve keyword extraction algorithms to achieve language independence in keyword extraction.

## Figures and Tables

**Figure 1:** Flow chart of clustering and keyword extraction method based on word vector.

**Figure 2:** The change curve of F-measure with the text-similarity threshold T.

**Figure 3:** Comparison of PRF values of different keyword extraction algorithms.

**Figure 4:** The results of different keywords extraction algorithms.

RETRACTED

**Table 1:** The result of text clustering.

Dataset	# Raw texts	# Extracted texts	Extraction ratio	## Feature words	Average word frequency of text	Coverage	F-measure
Data1	200	88	0.40	2400	92	0.88	0.89
Data2	400	270	0.60	5100	122	0.78	0.80
Data3	600	220	0.65	4800	126	0.77	0.72

## Data Availability

The data used to support the findings of this study are available from the corresponding author upon request.
